The article "Fears and Concerns of Bystanders to Help People Injured in Traffic Accidents: A Qualitative Descriptive Study" was published in 2023. Journal: Emerg Med Int.

# Fears and Concerns of Bystanders to Help People Injured in Traffic Accidents: A Qualitative Descriptive Study

**DOI:** 10.1155/2023/1862802

**Published:** 2023-12-07

**Authors:** Mohammad Jafar Sepahvand, Kian Nourozi, Hamidreza Khankeh, Farahnaz Mohammadi-Shahboulaghi, Masoud Fallahi-Khoshknab

**Affiliations:** ^1^Department of Nursing, University of Social Welfare and Rehabilitation Sciences, Tehran, Iran; ^2^Emergency and Disaster Health, University of Social Welfare and Rehabilitation Sciences, Associated at Department of Clinical Science and Education, Karolinska Institute, Tehran, Iran; ^3^Iranian Research Center on Aging, Nursing Department, University of Social Welfare and Rehabilitation Sciences, Tehran, Iran; ^4^Department of Nursing, Iranian Scientific Association of Nursing, University of Social Welfare and Rehabilitation Sciences, Tehran, Iran

## Abstract

In most traffic accidents, bystanders arrive at the scene before the rescuers. If they provide the right help, they can play an important and effective role in reducing the number of deaths and complications caused by these accidents. However, in many cases, fears and concerns prevent bystanders from providing assistance. This study aims to investigate and understand the fears and concerns of bystanders when they decide to help in traffic accidents. In 2022, this study was carried out in Iran using a qualitative content analysis approach. The data was collected through semistructured interviews. Participants were 15 males and females who had experience providing assistance in traffic accidents. Interviews, after digital recording, were transcribed verbatim. A purposeful and theoretical sampling method was performed. Data analysis and the determination of codes, categories, and subcategories were done using qualitative analysis software. O'Brien's qualitative research reporting standard was used. The results of the study include a category of fears and concerns and five subcategories. The subcategories include fear and concern caused by lack of information, fear of legal troubles, stress caused by previous experience, fear and anxiety caused by anticipation, and anxiety of unknown origin. The results of this study showed that some of the fears and concerns of the bystanders were related to a lack of information about providing assistance. By increasing bystanders' information about assistance, such as first aid training, fear and anxiety caused by a lack of information can be reduced. Another part of the fear and concern of bystanders is due to legal issues. Passing and implementing laws that protect bystanders can help reduce this fear and concern. Bystanders should be trained to provide assistance according to the rules of assistance so that they do not get into legal problems. A part of the bystander's fear and concern stems from their previous experiences providing assistance in traffic accidents. These experiences can also affect the fear and anxiety caused by anticipation. It is necessary to conduct more studies on the role of bystanders' experiences in creating fear and anxiety in them, as well as their effect on anticipatory fear.

The article "Fears and Concerns of Bystanders to Help People Injured in Traffic Accidents: A Qualitative Descriptive Study" was published in 2023. Journal: Emerg Med Int.

## 1. Introduction

Traffic accident injuries are the eighth leading cause of death in all age groups [1]. Providing help in the first few minutes of the accident is important [2–4]. In 85 to 97 percent of these accidents, bystanders arrive on the scene within the first few minutes after the accident [5, 6]. In only 11% of cases, they provided first aid [7], and in 68% of cases, they did not take any action and just watched the scene [7]. One of the important reasons for the lack of participation of bystanders in providing help is their fear and concern about helping out [8–10].

It is common for bystanders to experience fears and concerns during assistance [11]. Many mental and emotional factors affect their fears and concerns. The personalities of the bystanders and the circumstances of the incident can affect these factors [12]. Human behavior in social environments and conditions is different due to differences in the ability to learn, perceive, and interpret stimuli as well as their natural tendency to help [7, 13]. Bystanders act based on the representation, interpretation, and perception they have of reality, not on reality itself. Mental states such as intentions, beliefs, and desires have roles [13]. In addition to these, a set of situational and sociological factors affect the decision-making and performance of bystanders [14]. Care management at the scene of an accident is different from treatment environments such as hospitals. Also, facing many challenges, such as the unpredictable characteristics of the injured, emergency conditions, and the need to make quick decisions, can be effective. Panic, shock, and disbelief; conflicts requiring moral decisions [15, 16]; and anxiety [17] affect the way bystanders perceive and experience these fears and concerns. As a result, it affects the way bystanders make decisions to help [12, 13, 18].

While fears and concerns play a vital role in how bystanders make decisions to help victims of traffic accidents, there is limited information about them [8, 11, 19, 20]. By knowing more about the perspectives and experiences of bystanders in relation to fears and concerns and their related factors, it is possible to potentially improve guidelines [13, 21]. Knowing more about this phenomenon can also improve performance, confirm and support bystanders, reduce fear, and increase their participation in providing assistance [22]. For this purpose, this study was conducted with the aim of investigating the fears and concerns that influence the decisions of bystanders to provide assistance using the method of qualitative content analysis. Qualitative methods can play an important role in advancing the research agenda in emergency scenes. These kinds of studies allow researchers to gain a deep understanding of health problems or specific populations by examining the experiences and perspectives of participants [23].

The article "Fears and Concerns of Bystanders to Help People Injured in Traffic Accidents: A Qualitative Descriptive Study" was published in 2023. Journal: Emerg Med Int.

## 2. Materials and Methods

This study was conducted using the qualitative description method [24]. Data analysis was done by the content analysis method [25]. The participants are all lay people from different cities in Iran who witnessed the scene of a traffic accident and tried to help the victims of the accident. Entry criteria were to have experience providing assistance in traffic accidents, the ability to speak Persian, and the desire to participate in the study. People with expertise in the field of assistance who happened to be present at the scene of the accident could also participate in the study. Sampling was done purposefully, and in the continuation of the research, theoretical sampling was done.

### 2.1. Data Collection

In-depth, semistructured interviews with open-ended questions based on an interview guide (Table 1) were used to collect data. Such questions included, “If you have ever witnessed a traffic accident, please describe your experience.” Follow-up and exploratory questions were used. All interviews were conducted in Persian. Interviews were recorded by a digital audio recorder. All interviews were transcribed verbatim immediately after recording. The text of the interviews was entered into the qualitative analysis software MAXQDA2020. The duration of the interviews ranged from 30 to 60 minutes. The average was 45 minutes. The data collection spanned about two years, from April 2020 to April 2022. The data analysis was done simultaneously with their collection. The analysis of the text of the interviews was done in Persian. The results, codes, and classes from all the interviews were extracted in Persian and then translated into English. The number of participants until reaching conceptual saturation [26] was 15 (Table 2).

All interviews were conducted by the first author. He is a doctoral candidate in nursing education. At the doctoral level, he received the necessary training to conduct interviews and qualitative research. The researcher has certificates from workshops on data collection methods in qualitative research, proposal writing in qualitative research, and data analysis in qualitative research. All interviews were conducted with the guidance and supervision of other authors, who are all experienced professors in the field of conducting qualitative research.

The article "Fears and Concerns of Bystanders to Help People Injured in Traffic Accidents: A Qualitative Descriptive Study" was published in 2023. Journal: Emerg Med Int.

The start of sampling in this research almost coincided with the start of the spread of the COVID-19 disease around the world. The research team tried to conduct sampling and interviews in such a way that the participants as well as the research team did not pose a risk of getting infected. On the other hand, the participants were afraid of conducting face-to-face interviews. This caused the sampling process to be slow, especially in the first six months of the pandemic. After that, the research team decided to conduct some interviews by phone in order to protect the rights and health of the participants and members of the research team. With the passage of time, the scientific knowledge of the research team about COVID-19 increased. The research team took into account all the necessary health protocols to prevent disease transmission. We respect the rights of the participants, and if they agreed, nine interviews were conducted face-to-face.

At the end of each interview, the participant was asked if there was anything left to say about the incident he witnessed. He/she was also asked to mention if he had any suggestions to solve the problems he was facing. In the first 3 interviews, questions were asked based on the interview guide presented in Table 3. After that, due to the identification of some dimensions of fears and concerns, the process and type of questions changed a little. Then more focus was placed on finding the characteristics and dimensions of the fears and concerns found. Participants were chosen using theoretical sampling to assist in the development of less developed dimensions and characteristics of fears and concerns.

### 2.2. Data Analysis

Data analysis was done according to the steps proposed by Grandheim and Lundman [26]. With the permission of the participants, all interviews were recorded using a digital audio recorder. After the end of the interview, the audio file was listened to by the first author and transcribed verbatim. The similarity of the audio file of the interview with the transcribed text was checked. Then the text of the interview was entered into the MAXQDA software. The transcript file was provided to all authors. The interviews were coded separately by the first, second, and third authors. Disputed items were settled by consensus in the presence of all authors. After the consensus of all authors regarding the coding and analysis of each interview, based on the results obtained in each interview, the next interview was conducted. The interview guide was changed based on the results obtained in each interview. The first, second, and third authors did the coding simultaneously but separately with the help of the software. After coding each interview, the resulting files were shared. If there is a difference in the codes, a discussion and exchange of opinions were done in the presence of the fourth and fifth authors until reaching a consensus.

The article "Fears and Concerns of Bystanders to Help People Injured in Traffic Accidents: A Qualitative Descriptive Study" was published in 2023. Journal: Emerg Med Int.

The text of the interview was read once in its entirety to get a general picture of it in the author's mind. Then sentences or an entire paragraph of text were determined as units of meaning. Then, each sentence and each paragraph were read several times. By considering the mental states and feelings of the participants, the authors tried to extract the hidden content and symbolic meaning of the sentences. First, primary codes were extracted from them. Primary codes that were similar to each other or formed different dimensions of a concept were placed in one category by using the code creation part of the MAXQDA software. These categories formed the primary concepts. Similar primary concepts were combined into more comprehensive classes, and finally the hidden content and symbolic meaning in the data were determined.

After extracting the results, the results were shared with all participants, and they were asked to provide feedback on the results. They were also requested to suggest an appropriate solution to solve the problems found according to the study's results. The participants were asked to give a score from 1 to 10 to different challenges related to bystanders' fear and concern. 1 is the least fear and concern, and 10 is the most fear and worry. Based on the scores of the participants, the greatest fear and concern related to getting involved in legal issues and the fear of a lack of information to provide assistance were determined. Participants suggested reducing these fears and concerns by teaching first aid to community members and educating everyone in public media.

### 2.3. Trustworthiness

To validate the results, the following were done: Using an interview guide, allocating enough time to conduct interviews, continuous comparative analysis of data and classes in terms of similarities and differences, evaluation and confirmation of codes by other members of the research team, who were all expert professors in the field of conducting qualitative research, reaching a common consensus, checking and confirming the findings by several contributors, and long-term engagement with the data. The results of this research were reported using the O'Brien standard [27].

The article "Fears and Concerns of Bystanders to Help People Injured in Traffic Accidents: A Qualitative Descriptive Study" was published in 2023. Journal: Emerg Med Int.

### 2.4. Ethical Considerations

This study is part of the results of the Doctorate in Nursing thesis entitled “Explaining the decision-making process of bystanders to provide assistance in traffic accidents.” All research stages are supervised and coordinated by the Research Ethics Committee of the University of Social Welfare and Rehabilitation Sciences, with IR code USWR. REC.1398.023. Therefore, all participants voluntarily participated in the study; explaining the purpose and method of the study comprehensively to the participants; understanding the participants about the possibility of withdrawing from the study at any stage they wish; reading and signing the informed consent form by the participants; obtaining permission from the participants to record the interviews; ensuring the confidentiality of information in all stages of the research; and publishing the results are among the ethical considerations that were followed in this study.

## 3. Results

There were 15 participants, ten of whom (66%) were men and five (34%) were women. Nine interviews were conducted face-to-face, and Six interviews were conducted over the phone. The average age of the participants was 37.83 years, and their age range was from 28 to 52 years. Other demographic characteristics of the participants are presented in Table 2.

### 3.1.  Fears and Concerns

Based on the results of this study, fears and concerns include the following subcategories: fear of legal trouble, stress caused by previous experience, fear and concern caused by anticipation, fear and concern due to lack of information, fear and concern related to the relief forces, and concerns of unknown origin (Table 3).

#### 3.1.1.  Fear of Legal Problems

This fear may be due to previous legal problems or a lack of knowledge about the law of helping. The previous experience of legal trouble is the experience that the bystander has directly gained or that he or she predicts by knowing the experiences of other people or the media.

Participant #2: *“That's what I was thinking.” I thought that I was alone and that none of these people here would help me. And if something were to happen to that gentleman, everyone would be able to see that I went to him. Before the medical personnel arrive, call an ambulance and dial 115. I touched him. Now, if I touched him and he had a fracture or if it was possible to cut his spinal cord or put him in a bad position, then it was me. The responsibility was mine. “This would have affected me a lot.”*

The fear of not having enough information about laws can be due to a lack of training, insufficient training, or a lack of stability in the laws related to assistance. The fear of being accused is another fear related to the fear of legal trouble. In this case, the bystander is worried about being accused by other witnesses, injured relatives, or legal authorities of being the cause of the accident or of causing more damage to the injured person.

The article "Fears and Concerns of Bystanders to Help People Injured in Traffic Accidents: A Qualitative Descriptive Study" was published in 2023. Journal: Emerg Med Int.

Participant number 7: *“I think people don't help because they are afraid of the consequences, and they don't have much knowledge about how to help properly.” In the aforementioned accident, many people said, “Don't touch it; it might move badly, and the problem will get worse,” or something to that effect, but he said, “If I help, the really bad guy might escape, and they will catch me.”*

#### 3.1.2. Stress Caused by Previous Experience

Fear and concern in bystanders are caused by the information and experiences they have in relation to providing assistance. For example, if a bystander in the previous incident witnessed that another bystander, by providing incorrect assistance, caused more injuries and problems for the injured, in the current incident he or she may be fearful and concerned by observing the gathering of bystanders and seeing similar conditions. In this case, the source of fear and concern is mainly the bystander's own experiences and not the way other bystanders act.

Participant No. 8: *“At that moment, I wasn't really afraid, but I was anxious and worried.” I was worried that they wouldn't move the injured man. We already had several other cases in the family where people were moved and their spinal cords were severed. “It was, and I was very stressed about this.”*

#### 3.1.3. Fear and Concern Caused by Predicting

The fear and concerns of the bystander are related to the predictions that the bystander himself makes regarding the conditions and situations that may occur. These predictions can be related to dangers, such as the fear of an explosion, that the bystander knows about and predicts will happen. Although this explosion may never happen, the fear of its occurrence can affect how a bystander decides to help. In some cases, it may even cause the bystander to decide not to help.

Participant No. 1: *Participant No. 1: “I was thinking about not taking one of them out, and the car would explode before the other injured person got out. I was constantly thinking about these things. For example, the injured woman might come out and the injured man would remain. The father might die, and the child would become an orphan. In the few minutes I was knocking on the door, I was talking to the driver and thinking about these things at the same time.”*

#### 3.1.4. Fear and Concern due to a Lack of Information

In order to make a rational decision, the bystander must have some necessary information to decide. In the event of an accident, for some reason, the bystander cannot get the necessary information. Some of these reasons include the suddenness of the accident, not having enough time to decide, needing to act quickly and make quick decisions, and not having enough time or resources to get the required information. This lack of necessary information can cause fear, concern, and anxiety in the decision-maker. The fear and concern caused by the lack of information can also be caused by the fear of not checking the risks. In this case, the bystander did not check the risk of the accident scene due to reasons such as a lack of time, and this caused fear and concern in him.

The article "Fears and Concerns of Bystanders to Help People Injured in Traffic Accidents: A Qualitative Descriptive Study" was published in 2023. Journal: Emerg Med Int.

Participant No. 1: *“I said that I was a little scared because I didn't even look for a second to see if it was oil, gasoline, or whatever. But it was as if I heard them say that it was gasoline, that it spilled on the ground, and that the car may explode at any moment. I decided to take them out before it exploded.”*

#### 3.1.5. The Stress of the Rescuers' Delay

The longer the rescuers arrive at the scene of the accident, the more concerned the bystanders are, and they may feel more responsible for providing help. This stress may be caused by the delay of the rescue forces due to the bystander's perception that the rescue forces are late. In this case, even though the emergency services arrive at the scene of the accident at a reasonable time, the bystander imagines that they are delayed. This perception of delay causes stress and concern for the bystander.

Participant No. 11: “*I really don't know why I had pressed my fingers so hard on my palm; maybe for a day or two, the marks of my nails were on my palm because of the anxiety I felt because of the late arrival of these [rescue forces]*.”

#### 3.1.6. Anxiety of Unknown Origin

Part of the fear and concern of the bystanders may be due to reasons that are not known to the bystanders themselves. Traffic accidents are stressful by nature. This can cause a bystander to feel fear and concern even without a known reason, which can be called anxiety in this case and whose origin is not known. This anxiety can cause the bystander to unconsciously decide and act on some issues. In this case, the reason for that decision is not clear to the bystander himself.

## 4. Discussion

According to the findings of this study, one of the bystanders' fears and concerns in providing assistance is the fear of getting into legal trouble. Part of this fear is due to a lack of knowledge about the laws related to aid delivery. This can be caused by a lack of education, a lack of stability in the law, multiplicity, and diversity in the laws and law-making organizations. Another part of the fear of legal trouble is the fear of being accused; in this case, the person is afraid of being accused and sued for participating in helping. These results are similar to those of other studies [28–30]. In Hall's study, one of the important factors of fear in providing help in emergency situations is the fear of legal consequences and being sued. Hall's study showed that this fear increases when the person receiving help is a stranger and has no relationship with the bystander [11].

The article "Fears and Concerns of Bystanders to Help People Injured in Traffic Accidents: A Qualitative Descriptive Study" was published in 2023. Journal: Emerg Med Int.

In most similar studies, having previous experience providing assistance is considered a factor in increasing one's self-confidence and the ability of bystanders to help. Lack of experience providing assistance is regarded as a factor that increases bystanders' fear and concern to assist [11, 30]. Furthermore, the findings of other studies have shown that not having prior experience providing assistance can cause people to be unsure of what to expect at the scene of an accident and whether or not they can provide appropriate intervention [11]. The results of the present study, in addition to confirming these results, show that some experiences of witnesses in providing previous assistance can increase the incidence of fear and anxiety in order to provide assistance in the current incident. This requires further study.

In the fear and concern caused by predicting, the problem that the bystander is afraid of happening has not yet happened. The bystander predicts that the problem will happen according to the existing conditions. This prediction fills him or her with dread. Several studies have shown that predicting the occurrence of possible dangers and issues can cause the witness to decide not to help [8, 31, 32]. The results of the present study also show that these predictions may, in some cases, reduce the willingness of bystanders to help. Furthermore, in some cases, depending on the circumstances of the accident and the injured, they may cause the bystander to prevent the occurrence of the issues that he has predicted and take action to help.

In the fear and concern caused by a lack of information, the origin of it is a lack of information regarding the issue bystanders want to decide about. The results of other studies in this field are consistent with the results of the present study. Moreover, other studies show that if the first aid trainings are better, more qualitative, and more practical, and the bystander is more proficient in their implementation, these fears and concerns are reduced at the time of decision-making. In this situation, the willingness of bystanders to help will increase [10, 33]. Fear and concern about further harming the victim, leading to litigation, have been identified in many studies as barriers to the decision to provide assistance. It appears that bystanders who lack confidence in their knowledge of first aid do not consider themselves competent to help and are therefore less willing to help [8, 32]. Moreover, when the bystander is afraid of doing the wrong thing or of causing more harm, there is mainly a fear of legal conflicts [11, 34]. Part of this fear and concern can be attributed to a lack of knowledge about the laws that protect bystanders who want to help [35–37].

The article "Fears and Concerns of Bystanders to Help People Injured in Traffic Accidents: A Qualitative Descriptive Study" was published in 2023. Journal: Emerg Med Int.

The results of our study showed that a part of the fear and concern of the bystanders was due to a lack of information. This lack of information may be related to assistance information or a lack of information related to legal issues. Lack of information can reduce the willingness of bystanders to help because they fear that, due to not having enough information, they will cause more harm to the injured or that they will have legal problems. Other studies have also shown that sometimes bystanders do not intervene at the scene of an accident out of fear of not being able to help the injured person. Fear of doing the wrong thing, usually due to a lack of first aid training, is one of the most common reasons why bystanders refrain from taking lifesaving measures for the injured [7]. People experience a sense of uncertainty in emergency and unexpected situations [38–41]. This sense of uncertainty is caused by the lack of information [39, 40]. This uncertainty affects how they make decisions and help [39, 41]. Bystanders are afraid to ignore important information to save the victim's life [39]. Some people also fear legal consequences, criticism, or disciplinary actions [42].

The results of our study showed that, in addition to the lack of information, sometimes having some information and experiences can also cause fear and concern. If a person has had an unpleasant experience in his previous experience of helping, this experience can cause fear and concern in the next helping. This unpleasant experience can be related to mistakes in assistance, the behavior and performance of other bystanders, or legal problems. The personal experiences and beliefs of participants are known as a lens for understanding situations and affect their willingness to help [38, 43]. Differences in personal experiences can cause people to not always agree with other people's decisions. In Anderson et al.'s study, a number of more experienced participants stated that, in some cases, their experience indicated that they should refrain from performing resuscitation and stop providing aid. These individuals expressed frustration that other colleagues initiated or continued resuscitation efforts in such situations [43].

The article "Fears and Concerns of Bystanders to Help People Injured in Traffic Accidents: A Qualitative Descriptive Study" was published in 2023. Journal: Emerg Med Int.

Although the results of our study showed that a part of the fear and concern of bystanders is due to the lack of information regarding legal issues, the results of other studies have shown that even in situations where there are rules and guidelines for helping and people are aware of them, the conflict between these guidelines and the ethical standards of the helping person or the wishes of the patient may cause bystanders to not act according to instructions [39, 44, 45]. Correct ethical decisions may sometimes lead to deviations from guidelines or laws [42, 45]. Reforming laws on assistance and passing laws that protect bystanders can reduce the fear and concern caused by laws [46, 47].

There is literature on where bystander training happens. Bystander training can occur in a variety of settings, including schools, workplaces, and community centers [7, 22, 48]. The specific location of the training will depend on the target audience and the goals of the training program. For example, training for school-aged children may take place in schools, while training for adults may take place in workplaces or community centers. Some training programs may also be delivered online or through mobile applications. The effectiveness of bystander training programs may depend on factors such as the content of the training, the delivery method, and the level of engagement and participation from the trainees [49, 50].

## 5. Conclusion

According to the results of this study, a major part of the bystanders' fears and concerns are due to their lack of information regarding how to provide help as well as the laws related to providing help. This can be reduced by providing practical and appropriate training. The fear of legal trouble is one of the reasons for fear and concern among bystanders. Lack of legal information, a lack of up-to-date information about existing laws, a lack of bystander protection laws, and bystanders not being aware of the protection law are some of the things that cause this fear and concern. In the bystanders' previous experiences, the type and manner of the bystander's experiences, the mental point of view, and the way of perceiving and interpreting the conditions of the injured and the incident have a significant impact on fear and concern. Therefore, it is suggested that in the training of first aid courses, the previous experiences of bystanders and how those experiences influence their decision-making should be included in the training. Another part of fear and concern comes from anticipation. It seems that the bystander's previous experiences affect his or her prediction of possible future dangers. Therefore, it is proposed that in future studies, with quantitative research and questionnaires, the experiences of bystanders who have experience providing assistance should be identified and taught to other people in helper training programs. If people know the experiences and perceptions of a bystander at the time of providing assistance, they can better meet their need for knowledge and advice during training.

The article "Fears and Concerns of Bystanders to Help People Injured in Traffic Accidents: A Qualitative Descriptive Study" was published in 2023. Journal: Emerg Med Int.

### 5.1. Relevance to Clinical Practice

The results of this research increase the knowledge of bystanders' fears and concerns about providing help. This recognition can be used to reduce the fears and concerns of bystanders in providing assistance, increase their participation in providing assistance, and, as a result, reduce deaths and complications caused by traffic accidents.

### 5.2. Limitations

Considering that the scene of a traffic accident is stressful for bystanders and participating in providing assistance can create risks for these people, these factors can cause bias in witnesses' memories. To reduce the effect of memory bias, we tried to focus on the experiences of bystanders rather than the exact details of what happened in this study. Due to the spread of the COVID-19 virus, access to the participants was more limited, and to protect their health, some interviews were conducted over the phone.

## Figures and Tables

**Table 1:** Guide to conducting the interview.

No	Basic interview questions
1	Can you tell me about the accident you witnessed?
2	How did you decide to help?
3	What assistance did you do?
4	What fears and concerns influenced your decision at that moment?
5	What happened after this incident?
6	If you witness an accident again, how do you think you would make a decision?
7	What problems did you have in providing help?
8	If there were no problems, how would you make a decision?
9	What suggestions or solutions do you have to solve these problems?

	Follow-up questions

1	If you want to remember that incident, the moment you were... (For example, fear, worry and...) what were you thinking?
2	Tell me, how did it affect you?
3	What happened after that?
4	Please explain to me what you are saying
5	Can you tell me how it happened?
6	Can you tell me what that feeling was like?
7	Can you tell me what you saw?
8	Can you explain to me more about......?
9	Can you tell me what you mean by...?
10	Can you explain ...... more?
11	What do you think could prevent you from helping?
12	Is there anything left that you would like to tell me about this incident?

The article "Fears and Concerns of Bystanders to Help People Injured in Traffic Accidents: A Qualitative Descriptive Study" was published in 2023. Journal: Emerg Med Int.

**Table 2:** The demographic characteristics of the participants.

Number	Age (year)	Sex	Education	Job	Interview type
1	33	Male	Junior high school	Self-employment	Face to face
2	33	Female	Bachelor of science in nursing (BSN)	Nurse	Face to face
3	43	Male	Mechanic engineering	Oil company	Face to face
4	43	Male	Master of laws (LL.M)	Lawyer	Face to face
5	39	Female	Bachelor of disaster relief	Teacher of rescue and emergency medical courses	Telephone
6	28	Male	Diploma	Server	Face to face
7	28	Male	Bachelor of statistics	Food industry factories	Telephone
8	29	Female	Bachelor of general psychology	Hospital counseling center	Telephone
9	52	Male	Master of management	Road construction company	Telephone
10	37	Male	Bachelor of accounting	Accountant	Face to face
11	43	Female	Master of public administration (M.P.A)	Quality assurance manager of airport	Face to face
12	46	Male	Master of applied hydrology	Meteorological organization employee	Telephone
13	42	Male	Diploma	Practical nurse	Face to face
14	37	Female	Diploma	Housewife	Telephone
15	47	Male	Diploma	Worker	Face to face

**Table 3:** “Fear and concerns” with subcategories and open codes.

Category	Subcategory	Open codes
Fears and concerns	Fear of legal trouble	Fear of being accused
		Previous experiences with legal trouble (direct experiences from the helper herself or himself; get experiences from other people; get experiences from the media)
		Lack of information regarding aid laws (lack of stability in aid rules), (not receiving training about the rules of giving aid)
	Stress caused by previous experience	The stress caused by the bystander gathering
		Concerned about the gathering of bystanders
	Fear and concern caused by anticipation	Concern about an unfortunate incident
		Fear of potential dangers
		The fear of an explosion
		Concern for the lives of the victims of the accident
		Predicting the situation to worsen
		Helping consequences (considering financial consequences), (considering helping consequences)
	Fear and concern caused by a lack of information	Fear of making a mistake
		Fear of causing more damage
		Uncertainty about the death of the injured
		Not knowing the number of injured
		Fear of not checking the risks
	Fear and concern related to the relief forces	The stress of delaying rescuers
	Concerning an unknown origin	Behaving instinctively

## Data Availability

The data that support the findings of this study are available upon request from the corresponding author. The data are not publicly available due to restrictions e.g., their containing information that could compromise the privacy of research participants.

## Additional Points

What is known or added. The results of this research can be used to reduce the fears and concerns of bystanders in providing assistance, increase their participation in providing assistance, and, as a result, reduce deaths and complications caused by traffic accidents. The results of this study will increase the knowledge of nurses and other global clinical communities about how to behave and help bystanders at the scene of traffic accidents. The source of information collection for this research was people from the community who were present at the scene of the accident as bystanders and had provided assistance. These people include both lay people of the society and people who are experts in the field of assistance. Reporting Method. EQUATOR guidelines called SRQR were used to report the results of this research.
